# A Research Study to Measure the Efficacy of Terminating Cervical Cancer via Customized Optimum Pathway

This article has been retracted.

**DOI:** 10.1155/2022/7872915

**Published:** 2022-03-15

**Authors:** Xianyu Zhang, Huan Ma, Xiurong Lu, Zhilin Zhang

**Affiliations:** Department of Radiotherapy, The First Affiliated Hospital of Hebei North University, Zhangjiakou, Hebei, China

## Abstract

**Background:**

To develop a precise prognostic model of overall survival in patients with terminating cervical cancer based on surveillance, epidemiology, and end results (SEER) program.

**Methods:**

The patients were retrieved from SEER data who are diagnosed with terminating cervical cancer from 2004 to 2016. The data were performed using univariate and multivariate analyses and constructed nomograms for predicting survival. Use C-index to validate the model accuracy.

**Results:**

Totally 15839 patients diagnosed with cervical cancer were independently allocated into the training set (*n* = 11088) and validation set (*n* = 4751). The multivariate analysis results indicated that age, race, stage_T, stage_M, and stage_N were confirmed as independent risk predictors, and those factors are applied to construct this clinical model. The C-index of overall survival in the training set was 0.6816 (95% confidence intervene (CI), 0.694–0.763) and that in the validation set was 0.6931(95% CI, 0.613–0.779). All calibration curves of various factors were consistent with predicted and actual survival.

**Conclusion:**

The nomogram provides a novel method for predicting the survival of patients with terminating cervical cancer, assisting in accurate therapeutic methods for patients with primary terminating cervical cancer.

## 1. Introduction

Cervical cancer is the most common malignancy in female genital tract [1]. The incidence rate of cervical cancer is second in women and even in some underdeveloped countries and regions [2, 3]. The latest data show that there are about 500000 new cases of cervical cancer worldwide every year, of which more than 80% are in developing countries [4]. More than 260000 women die of cervical cancer every year, mainly in low and middle-income countries [5]. In China, the incidence rate of cervical cancer accounts for 11.9% of the total worldwide, and the death rate accounts for 11.1% [6]. The age of onset is younger. At present, gene expression microarray has been widely used to study gene expression profile [7]. Gene expression microarray is a credible and high-efficiency way to identify target genes. These microarray spectra not only provide a new method for studying various disease-related genes but also provide a good prospect for molecular prediction, drug-based molecular targeting, and molecular therapy [8, 9]. With the wide application of gene expression chip technology, a large number of data are published on the public database platform [10]. Using these databases can further study the molecular mechanisms related to diseases [11].

Nomograms have been applied on various disorders [12–16], and surveillance, epidemiology, and SEER data served as an all-around database to search cancers. By using all-around SEER database to assess different factors, the nomograms could predict survival prognosis [17]. Nomogram is a mathematical model based on multivariate regression analysis. Through this model, a variety of independent prognostic factors can be gathered together to make the predictive value more individualized and intuitive [18, 19].

In our study, we develop a precise prognostic model of overall survival in patients with terminating cervical cancer based on surveillance, epidemiology, and end results (SEER) program, which aimed to help clinical patients to relieve their disease.

## 2. Materials and Methods

### 2.1. Patients and Ethic

The patients were retrieved from the SEER data, which included information related to cancer prevalence, incidence, race, histological types, pathological types, survival time, and treatment at 18 registries in the USA. All the participants were diagnosed with cervical cancer by histopathological examination. The experiments were approved by the clinical research ethics committee hospital. All patients wrote the informed consent, in accordance with the provisions of the Helsinki Declaration of 1975.

Inclusive standard: patients were diagnosed with cervical cancer by histopathological means, age ≥18 years old, and patient's clinical information is complete.

Exclusion criteria: patients were with more primary carcinomas or secondary tumor and data about survival time or other clinical characteristics were missing.

### 2.2. Study Variables

The basic patient data were collected. The survival time (1 year, 3 years and 5 years) is related to invasive depth of tumor (T stage) (1 = T0, 2 = T1, 3 = T2, 4 = T3 and T3a and T3b, 5 = T4 and T4a and T4b, and 6 = TX), the number of involved lymph node (N stage) (1 = N0, 2 = N1, 3 = N2, 4 = N3, and 5 = Nx), and distant metastasis (M stage) (1 = M0, 2 = M1).

### 2.3. Construction and Validation of the Nomogram

All statistical data were conducted using R software 3.3.0 (R Foundation for Statistical Computing, Vienna, Austria, www.r-project.org). Second, we constructed a nomogram used the multivariate Cox regression-the area under the curve (AUC) by R software to confirm the factors; furthermore, we used concordance index and calibration curves to assess the accuracy. The Kaplan–Meier method is applied to verify the accuracy of survival curves [20]. The prognostic value of the factors was confirmed by Cox regression analyses [21]. Value of *P* < 0.05 was considered statistically significant.

### 2.4. Statistical Analyses

The data were compiled using with SPSS 19.0 statistical software. Values are presented as means ± SEM. The results were compared using Student's *t*-test. Kaplan–Meier survival analyses were used to analyze the clinicopathologic features. All experiments were performed in triplicate and a *P* value.

## 3. Results

### 3.1. Clinicopathological Characteristics of the Training and Validation Sets

Totally, 15839 qualified subjects were independently allocated into the training group (*n* = 11088) and validation group (*n* = 4751). As given in Table 1, there was no statistical significance between two groups in race, age, stage_T, stage_N, and stage_M (*P* > 0.05).

### 3.2. Survival Analysis in the Training Set

As shown in Figure 1, age, stage_T, stage_N, and stage_M were significantly associated with overall survival (OS) in Kaplan–Meier mean.

### 3.3. Prognostic Factors in the Training Set

Univariate analysis and multivariate analysis are given in Table 2. The results showed that factors such as age, race, invasive depth of tumor (T stage), the number of involved lymph node (N stage), and distant metastasis (M stage) were related to survival time. Mostly, stage_T, stage_N, and stage_M were important factors. Furthermore, we did further analyze binary logistic regression analysis to identify factors potentially predict cervical cancer development. Race, stage_T, stage_N, and stage_M were conformed as independent predictors for individual with cervical cancer.

### 3.4. Construction of the Nomogram

The nomogram was constructed by collecting all independent predictors for OS in the training cohort [22]. The model indicated that age ≧70 years old was most associated with survival for individual with cervical cancer, followed by TX stage and distant metastasis. Race and NX had moderate impacts on survival outcomes (Figure 2).

### 3.5. The Internal Validation of Nomogram

The nomogram had an exact prediction in cervical cancer development, and the unadjusted concordance index in the training set showed 0.6816 (95% CI, 0.694–0.763) and that in the validation set was 0.6931 (95% CI, 0.613–0.779). It indicated that the nomogram precisely predicts OS. Area under the curves (AUCs) are used to predict overall survival at 3 years and 5 years using the internal validation cohort (Figure 3). The 3 years and 5 years of AUCs were, respectively, 0.758, 0.788, and 0.792. This indicated that this nomogram model had a good predictive performance.

### 3.6. The External Validation of Nomogram

The external validation set result demonstrated that the model was exact. As shown in Figures 4 and 5, the proper consistency is between the predicted and observed OS for 3 and 5 years.

## 4. Discussion

Cervical cancer is one of the three most common gynecological tumors and has become the fourth leading cause of cancer-related death in women all over the world. Early screening and prevention of cervical cancer are of great importance in reducing the incidence rate and mortality of cervical cancer in China. Therefore, it is still worth to explore the pathological mechanism and find the genes related to the development of cervical cancer.

In our study, 15839 subjects were retrieved from the SEER data and construct the survival prognosis model. Age, race, stage_T, stage_N, and stage_M were confirmed as the independent prognostic factors. The nomogram displays a comparably higher C-index value and calibration, which indicated that it had a better appraise survival prediction performance.

The nomogram model contains more prediction factors, so that it has higher prediction accuracy than the traditional staging model [23]. In our study, a nomogram was developed with 15839 patients which is based on the SEER database, and we predicted that the overall survival time relied on the independently factors: age, race, stage_M, stage_N, and stage_T.

This research has some limitations. First, the nomogram model is based on the SEER database. Although the database covers 28% of the population in the United States and collects clinical data from multiple medical centers in the United States, it lacks some information, for example, treatment details and so on. Second, this study confirmed that the prognosis of cervical cancer patients is related with metastasis sites, but the SEER database only contains four specific distant metastasis sites. However, adrenal metastasis is also one of the common metastasis sites of cervical cancer, and this part of data is lacked in the database, which will affect the result of prognosis. Third, the nomogram model is based on the SEER database, which mainly collects clinical information of Western patients; the number of patients in the validation cohort is small. Therefore, a larger sample size of external data is needed for further validation to verify the credibility and universality of the nomogram model.

## 5. Conclusion

The nomogram provide a novel method for predicting the survival of patients with terminating cervical cancer, assisting in accurate therapeutic methods for patients with primary terminating cervical cancer.

## Figures and Tables

**Figure 1:** Kaplan–Meier survival curves for overall survival in the training cohort as stratified by (a) age, (b) race, (c) stage_T, (d) stage_M, and (e) stage_N.

**Figure 2:** Area under the curves to predict overall survival at 3 years (a) and 5 years (b) using the internal validation cohort.

**Figure 3:** (a) Te calibration curves for predictions of overall survival in the training set at 3 years and (b) 5 years after diagnosis. Te dashed line represents perfect agreement between the nomogram-predicted probability (*x*-axis) and the actual probability, calculated from a Kaplan–Meier analysis (*y*-axis).

**Figure 4:** (a) Te calibration curves for predictions of overall survival in the validation set at 3 years and (b) 5 years after diagnosis. Te dashed line represents perfect agreement between the nomogram-predicted probability (*x*-axis) and the actual probability, calculated from a Kaplan–Meier analysis (*y*-axis).

**Figure 5:** Nomogram predicting 3 and 5-year overall survival for patients with cervical cancer.

**Table 1:** Clinicopathological characteristics of the training and validation sets.

	Training set (*n* = 11088)	Validation set (*n* = 4751)	*P* value
Age (years)			0.584
<50	8425 (76%)	3515 (74%)	
50–69	1774 (16%)	730 (15.4%)	
≧70	889 (8%)	506 (10.6%)	

Race			
White	6376 (57.5%)	2755 (58%)	
Black	3060 (27.6%)	1235 (26%)	
Others	1652 (14.9%)	761 (16%)	

Stage_T			0.196
T0	3880 (35%)	1615 (34%)	
T1	3215 (27%)	1377 (29%)	
T2	2106 (19%)	997 (21%)	
T3	887 (8%)	332 (7%)	
T4	665 (6%)	237 (5%)	
TX	665 (5%)	157 (4%)	

Stage_M			0.881
M0	8532 (77%)	3563 (75%)	
M1	2556 (23%)	1188 (25%)	

Stage_N			0.304
N0	4546 (41%)	1852 (29%)	
N1	3659 (33%)	1615 (34%)	
N2	1108 (10%)	855 (18%)	
N3	1219 (11%)	570 (12%)	
NX	665 (5%)	332 (7%)	

*P* < 0.05, significant difference.

**Table 2:** Risk factors for OS according to the Cox proportional hazards regression model.

	Univariate analysis			Multivariate analysis		
	HR	95% CI	*P* value	HR	95% CI	*P* value
Age (years)						
<50	Reference					
50–69	1.3174	1.1744–1.4778	<0.001	1.2767	1.1593–1.4060	<0.001
≧70	1.7925	1.5980–2.0108	<0.001	1.7058	1.5491–1.8784	<0.001

Race						
Black	Reference					
White	1.7911	0.9266–1.0537	<0.001	0.9952	0.9435–1.0497	<0.001
Others	0.9881	0.7178–0.8719	0.7142	0.8000	0.7375–0.8677	0.85994

Stage_T						
T0	Reference					
T1	0.9497	0.5843–0.9619	0.0235	0.7225	0.5844–0.8932	0.00266
T2	1.0924	0.8552–1.3953	0.0193	1.0626	0.8627–1.3087	0.00323
T3	1.2169	0.9528–1.5542	0.1158	1.1750	0.9539–1.4474	0.12949
T4	1.2521	0.9810–1.5981	0.0710	1.2163	0.9880–1.4973	0.06487
TX	1.3546	1.0580–1.7344	0.0161	1.3164	1.0664–1.6249	0.01052

Stage_M						
M0	Reference					
M1	2.4121	2.3003–2.5293	<0.001	2.3545	2.2632–2.4495	<0.001
Stage_N						

N0	Reference					
N1	1.2549	1.1513–1.3678	<0.001	1.2307	1.1448–1.3231	<0.001
N2	1.3563	1.2851–1.4314	<0.001	1.3810	1.3199–1.4449	<0.001
N3	1.3033	1.2172–1.3954	<0.001	1.3537	1.2779–1.4341	<0.001
NX	1.3443	1.2324–1.4663	<0.001	1.3919	1.2932–1.4981	<0.001

*P* < 0.05, significant difference. HR, hazard ratio.

## Data Availability

The data used to support the findings of this study are available from the corresponding author upon request.
